# Secreted frizzled-related protein 5 promotes angiogenesis of human umbilical vein endothelial cells and alleviates myocardial injury in diabetic mice with myocardial infarction by inhibiting Wnt5a/JNK signaling

This article has been retracted.

**DOI:** 10.1080/21655979.2022.2070964

**Published:** 2022-05-04

**Authors:** Nian Ding, Chenghong Zheng

**Affiliations:** a Clinical College of Traditional Chinese medicine, Hubei University of Chinese Medicine, Wuhan, China; b Medical Ward, Wuhan Hospital of Traditional Chinese Medicine, Wuhan, China

**Keywords:** SFRP5, HUVECs, diabetic myocardial ischemia mice, angiogenesis, myocardial injury

## Abstract

The purpose of this study is to investigate whether secreted frizzled-related protein 5 (SFRP5) affects the proliferation, migration and angiogenesis of human umbilical vein endothelial cells (HUVECs) induced by high glucose (HG). HUVECs were treated with different concentrations of glucose. MTT, wound healing, angiogenesis, and ELISA assays were used to detect cell cytotoxicity, migration, tube formation, and VEGF165 and VEGF165b levels, respectively. The mice model of type 2 diabetes mellitus (T2DM) complicated with myocardial infarction (MI) was established. SFRP5 was injected intrabitoneally for 2 weeks. cardiac output (CO), left ventricular ejection fraction (LVEF) and left ventricular shortening fraction (LVSF) were detected by echocardiography. Western blot was used to detect the protein levels of SFRP5, Wnt5a, JNK1/2/3, p-JNK1/2/3, TGF-β1, Caspase3, Bax, and Bcl-2. The expression of SFRP5 was declined in HG-induced HUVECs and T2DM-MI. Intervention of SFRP5 promoted the migration of HUVECs and angiogenesis, as evidenced by a lower expression of Bax and caspase3, but a higher expression of Bcl-2. Meanwhile, SFRP5 inhibition repress Wnt5a and p-JNK expression. Howerver, The JNK inhibitor (SP600125) enhanced the down-regulation of Wnt5a/JNK pathway proteins by SFRP5. SFRP5 intervention increased the levels of CO, LVSF, and LVEF in T2DM-MI mice. SFRP5 inhibited myocardial pathological injury and fibrosis in T2DM-MI mice and SFRP5 could down-regulate Wnt5a and p-JNK1/2/3 activation. SFRP5 promotes the proliferation, migration and angiogenesis of HUVECs induced by HG, and inhibits cardiac dysfunction, pathological damage, fibrosis, and myocardial angiogenesis in diabetic myocardial ischemia mice, which is achieved by inhibiting Wnt5a/JNK signaling.

## Research highlights

(1) HG reduced HUVECs activity, cytokine production, and angiogenesis

(2) SFRP5/Wnt5a/JNK axis activation reduced angiogenesis in HUVECs

(3) SFRP5 reduced MI in T2DM mice complicated with MI by repressing the Wnt5a/JNK pathway

## Introduction

Diabetes has become a global problem and threatens human health [1,2]. Beyond normal range, the blood sugar level is categorized into two categories as hyperglycemia (glucose concentration > 1.20 mg/mL) and hypoglycemia (glucose concentration < 0.80 mg/mL) [3]. Diabetic patients are characterized by elevated blood sugar levels, accompanied by multiple complications. These serious complications lead to higher disability and mortality [4,5]. Hyperglycemia damages nerve fibers, such as sensory nerve fibers, leading to painless myocardial infarction, reducing the synthesis and release of cardiac protective neurotransmitters, and further increasing the incidence of cardiovascular events and sudden cardiac death [6]. In addition, abnormal vascular endothelial cell function can cause diabetic angiopathy, and hyperglycemia can cause vascular endothelial cell injury and apoptosis [7,8]. Nevertheless, the mechanism of impaired endothelial function after diabetes and the mechanism of revascularization after ischemia are not yet fully understood.

Vascular endothelial cell injury is the initiating link and pathophysiological basis of diabetic angiopathy. Early effective intervention of HG vascular endothelial injury is of positive significance in preventing and treating diabetic vascular complications [9,10]. At present, the drugs or measures to block the progressive aggravation of endothelial injury are still in the exploratory stage. Epidemiological trends worldwide show that despite the very advanced treatment strategies for hyperglycemia, high blood pressure, and dyslipidemia, severe diabetic microangiopathy still exists. Endothelial cells play a very important role in maintaining and repairing angiogenesis, and their functions directly affect the development of diabetes [11–14].

Secret frizzled related protein 5 (SFRP5) is a Wnt signal suppressor protein, which regulates Wnt signal through direct interaction with Wnt. They play a role in regulating cell growth and differentiation of specific cell types [15–17]. Binbin Guan et al. Found that SFRP5 was markedly down regulated in primary mouse islet cells stimulated by HG. Increasing SFRP5 could inhibit the proliferation of primary mouse islet cells induced by HG, and inhibited the expression of Wnt signal pathway and cyclin CD2. They also found that HG inhibited the expression of SFRP5 protein through PI3K/Akt signal [18]. Carstensenkirberg M et al found that the high expression of SFRP5 protein was negatively correlated with the risk of type 2 diabetes and heart disease, indicating that SFRP5 could serve as a new target for cardiovascular disease [19]. Previous studies unanimously reported that SFRP5 exerted an anti-inflammatory effect by inhibiting the non-canonical Wnt5a/JNK signaling pathway, therefore playing a key role in repressing the occurrence and development of various diseases including obesity, cardiovascular diseases, and diabetes [20]. However, the function and mechanism of SFRP5 in diabetic injury need to be further elucidated.

We hypothesized that SFRP5 might play a potential role in T2DM angiogenesis and alleviate myocardial injury through certain mechanisms. In view of the above research basis, this study explored the role of SFRP5 in HG induced HUVECs and diabetic myocardial infarction, and confirmed that SFRP5 promoted HG induced HUVECs proliferation, migration and angiogenesis, and inhibited cardiac function impairment, pathological damage, fibrosis and myocardial angiogenesis by inhibiting Wnt5a/JNK signaling. This finding can provide some references for molecular targeted therapy in diabetes and its complications.

## Materials and methods

### Cell culture

Cell culture was performed as described previously [21]. HUVECs were purchased from American Type Culture Collection (ATCC, Manassas, Virginia). The cells were cultured in complete ECM medium (Hyclone; GE Healthcare Life Sciences, Logan, UT, USA) containing 5% FBS, 1% penicillin, and streptomycin (GIBCO, USA) were added, and cultured in a incubator at 5% CO_2_, 37°C. The cells of the 3rd–5th generation in logarithmic growth period were used for subsequent experiments. HUVECs were cultured at 37°C for 24, 48 and 72 h. ECM contained different concentrations of glucose (5, 11, 25, 30 mmol/L) to simulate HG.

### Cell transfection

Cells were transfected as described previously [22]. Took the cells cultured to logarithmic growth stage, changed the culture medium to the culture medium without fetal bovine serum (FBS) one hour before transfection, and transfected with reference to Lipofectamine 2000 transfection kit. SFRP5 negative control plasmid, si-SFRP5 and SFRP5 (100 nmol/L, Guangzhou Ruibo biology Co., Ltd.) were transfected into HG induced HUVECs, respectively. After 6 h of transfection, the culture medium was changed into full culture medium, cultured at 37°C, 5% CO_2_ for 48 h, and the cell supernatant was collected.

### MTT

Cellular proliferation was quantified as described previously [23]. Took logarithmic growth cells and adjusted the cell density so that the density to be measured was 5 × 10^3^ cells/well were inoculated into 96-well plates. After the cells adhered to the wall, low serum medium (2% FBS) containing different concentrations of glucose was added. Five multiple wells were set in each well. In addition, the medium without cells was set as the blank control and cultured in 37°C 5% CO_2_ incubator for different times, the cell fusion was observed under an inverted microscope, Added 20 μL MTT solution to each well, continued to culture for 4 h, carefully sucked out the culture medium in each well, added 100 μL DMSO to each well, shook on the shaking table at low speed for 5–10 min, and measured the absorbability of each well with a microplate reader (Bio-RAD Laboratories, Inc.) at wavelength 490 nm within 30 min. The experiment was repeated three times.

### Wound healing assay

Wound healing assay was carried out as we described previously [24]. Drew a horizontal line with a ruler behind the 6-well plates with a marking pen, and the horizontal line passes through the hole. Endothelial cells in logarithmic growth stage were divided into 2 × 10^5^ cells/well were inoculated in 6-well plates. On the next day, when the cells have grown to about 80% confluence, scratched with 10 μL microsample gun head perpendicular to the horizontal line on the 6-well plate. Washed it twice on PBS. Removed the floating cells from the scratch. The medium was replaced with 2% FBS and stimulated with different concentrations of glucose at the same time, so that the final concentration was 30 mmol/L. The scratch location was photographed for 0 h with a camera and recorded. The location was cultured in a 37°C, 5% CO_2_ incubator. The same location was photographed for 12, 24, and 48 h, and the scratch distance was measured with Image-Pro Plus. The experiment set up a compound hole, repeated three times, according to the cell crawling distance measurement of its migration ability.

### Enzyme-linked immunosorbent assay (ELISA)

Ninety-six-well plates were cultured in 5% CO_2_ and 37°C incubators for 48 h, respectively, and the cell supernatant was absorbed, respectively. The detection was carried out according to the operation instructions of the ELISA kit of vascular endothelial growth factor 165 (VEGF165) and VEGF165b (Tiangen Biotechnology Co., Ltd.). The ELISA was done as previously described [25].

### Tubule forming ability detection

In vitro angiogenesis (capillary tube formation assay) was performed as previously described [26]. Matrigel was thawed in the refrigerator at 4°C in advance, and the gun head box and 96-well plate were pre-cooled in the refrigerator at 4°C in advance. The thawed matrigel stock was added to the 96-well plates (50 μL/well), evenly paved, and placed in the incubator at 37°C with 5% CO_2_ for 30 min. Meanwhile, cell suspension was prepared. After the cells in the culture flask were digested, the cell density was adjusted to 1.5 × 10^4^, and the mixture of cell reagents of different experimental groups was prepared. The cells were evenly inoculated with 100 μL per well into a 96-well plate coated by matrigel. The cells were cultured at 37°C in 5% CO_2_ incubator for 7 h, and the formation of lumen was observed and took photos to record analysis.

### Western blot

Western blot was performed as described previously [27]. HUVECs were inoculated into 60 mmol/L culture dishes. When the adherent growth reached 80%, different treatment factors were given. The culture medium was discarded, washed twice with precooled PBS, and added 80 μL lysis solution to each dish and cook at 4°C for 30 min. Centrifugation at 12,000 r/min for 15 min, took the supernatant, and determined the protein concentration by BCA method. The total protein was separated by SDS-PAGE and transferred to PVDF membrane (Beijing pulley gene). Sealed with 5% skimmed milk powder for 90 min, and added various primary antibody SFRP5 (ab230425, 1:1000, Abcam), Wnt5a (ab282153, 1:500), p-JNK1/2/3 (ab124956, 1:1000), caspase3 (ab32351, 1:5000), Bax (ab32503, 1:1000), Bcl-2 (ab182858, 1:2000) and TGF-β1 (ab215715, 1:1000), 4°C overnight, then washed with Tris Buffered Saline with Tween (TBST) for 3 times (10 min each time), added secondary antibody (1:1000), incubated at room temperature for 60 min, and then washed with tbst for 3 times (10 min each time). The PVDF film was colored by ECL solution, exposed to darkroom, and analyzed by gel imaging system.

### Model preparation and SFRP5 intervention

A model of STZ‐induced diabetic mice was established as previously described [28]. All mice were purchased from the experimental animal center of Hubei University of Chinese Medicine. Forty male C57BL/6 mice (6–8 weeks of age) were selected. After adaptive feeding for 1 week, 10 mice were randomly selected as the normal group and given ordinary feed, and the rest were given high-fat feed. One month later, each group fasted for 12 h (overnight), the high-fat group received intraperitoneal injection of streptozotocin (40 mg/kg) after 4 weeks, and the normal group received the same volume of sodium citrate buffer. Another injection in 4 h, continuous 3 d, fasting blood glucose was more than 11.1 mmol/L, and the model of type 2 diabetes was successful. For the MI model, the procedure was followed as previously described [29]. Ten mice who met the criteria of diabetes model were randomly selected as control group. The rest were given intravenous anesthesia with pentobarbital sodium 50 mg/kg, and the electrocardiogram electrodes were subcutaneously attached to the operation table, and the standard II lead electrocardiogram was recorded. Endotracheal intubation and ventilator. Opened the chest at the left third intercostal space, cut the open-heart bag, exposed the heart, ligated 1/3 at the beginning of the anterior descending branch of the left coronary artery with 6–0 nylon suture, took up the suture and tied the knot after dozens of cardiac cycles, and determined the success of the model with pathological Q wave in ECG, unidirectional ST segment elevation, and inverted T wave as the index. After several minutes of observation, closed the chest layer by layer, placed a drainage tube in the incision, and pulled out the endotracheal intubation when the mouse’s spontaneous breathing recovers. The mice in the control group underwent sham operation and intramuscular injection of penicillin to prevent infection. The model mice were randomly divided into diabetic infarction group (T2DM + MI) and SFRP5 intervention group (T2DM + MI + SFRP5), with 10 mice in each group. In T2DM + MI + SFRP5 group, SFRP5 (20 μg/kg*d) was injected intraperitoneally for 2 weeks. Mouse VEGF concentrations were measured with the Mouse VEGF165 Quantikine ELISA Kit (EK-Bioscience) and Mouse VEGF165b Quantikine Kit (Bioswamp). The experimental animals were disposed in strict accordance with the ethical regulations of the experimental animal center of Hubei University of Chinese Medicine.

### Echocardiography

Echocardiography analysis was performed as described previously [30]. After operation 4 weeks, the structure and function of the left ventricle of each mouse were evaluated by noninvasive transthoracic echocardiography. In short, anesthetized mice evaluated the parameters of cardiac structure and function on two-dimensional ultrasound-guided m-curve. Cardiac output (CO), left ventricular ejection fraction (LVEF) and left ventricular shortening fraction (LVSF) parameters were recorded automatically. Aloca5000 color ultrasonic diagnostic instrument was used.

### Hematoxylin eosin (HE) staining

HE staining was carried out as previously described [31]. The apical myocardium of rats was soaked and fixed with 10% paraformaldehyde for 12 h, and the thickness was 3 ~ 4 μM tissue sections, washed with deionized water for 1 ~ 2 min, stained with hematoxylin for 50s, washed with deionized water again for 1 ~ 2 min, fixed in absolute ethanol (including 1% HCl) for 30s, stained with eosin for 6 ~ 8 s, washed with deionized water for 1 ~ 2 min, fixed in absolute ethanol for 3 min, embedded in paraffin, and observed and analyzed in 5 different visual fields.

### Masson staining

Masson staining was performed as previously described [32]. The dewaxed and dehydrated sections were treated with 1% hydrochloric acid solution for 3 ~ 5 s and then rinsed. They were dyed with mild alkaline fuchsin solution for 3 min, rinsed with deionized water, treated with 1% phosphomolybdic acid solution for 1 min. After removing the residual phosphomolybdic acid solution with deionized water, they were dyed with 2% aniline blue solution for 2 min, rinsed and dehydrated with 95% ethanol, and embedded after drying. After staining, myocardial collagen fibers were blue-green and myocardial tissue was red under light microscope.

### Statistical analysis

Statistical analysis was done as previously described [33]. The experimental data were expressed as mean ± SD and SPSS 20.0 statistical software for statistical analysis. SNK-q test (comparison between experimental groups) and dunnett-t test (comparison between experimental group and control group) were used. The difference was statistically significant (*P* < 0.05).

## Results

In this study, the regulatory effect of the SFRP5/Wnt5a/JNK signal axis on angiogenesis in T2DM was investigated. The expression of these proteins were detected in T2DM mice with MI and HUVECs induced by HG. In addition, proliferation and migration of HUVECs as well as degree of angiogenesis were investigated. We hypothesized that SFRP5 alleviates the angiogenesis of HUVECs, and mechanistically regulates Wnt5a/JNK signaling pathway.

## HG induced HUVECs activity, cytokine changes, and angiogenesis

HUVECs were treated with different concentrations of glucose (5.5, 11, 25, 30 mmol/L) for 24, 48, and 72 h, respectively, MTT assay showed that the cell activity of HUVECs treated with different concentrations of glucose decreased significantly in a time-dependent manner, indicating that HG increased endothelial cytotoxicity. The activity was lowest when the concentration of HG was 30 mmol/L for 72 h. According to the results of cell proliferation rate, 30 mmol/L HG for 72 h was selected as the best condition for the following experiments (*P* < 0.05, Figure 1(a)). The migration of HUVECs at 0, 12, 24, and 48 h was detected by scratch test at the optimal sugar damage concentration (30 mmol/L). The results showed that the migration distance of HUVECs in HG group was lower than that in NC group (*P* < 0.05, Figure 1(b)). Subsequently, ELISA results showed that compared with NC group, the expression of VEGF165 was up-regulated and VEGF165b was down regulated in HG group (*P* < 0.05, Figure 1(c, d)). Then, the tube forming ability of HUVECs induced by HG was detected, the results showed that more tubes and naked bodies were observed in the control group than in the HG group (*P* < 0.05, Figure 1(e)). This indicates that the level of angiogenesis is weakened under HG. In addition, the regulatory role of Wnt5a/JNK pathway in HG induced HUVECs was detected. Western blot results showed that the expressions of Wnt5a, p-JNK1/JNK1, p-JNK2/JNK2, p-JNK3/JNK3 were significantly up-regulated under HG conditions (*P* < 0.05, figure 1(f-h0)), indicating that Wnt5a/JNK pathway was involved in endothelial cell proliferation and angiogenesis.

**Figure 1.** HG induced HUVECs activity, cytokine changes and angiogenesis. (a) HUVECs were treated with different concentrations of glucose (5.5, 11, 25, 30 mmol/L) for 24, 48 and 72 h respectively. The activity of HUVECs was detected by MTT assay. According to the results of cell proliferation rate, HUVECs were treated with 30 mmol/L HG for 72 h, (b) The migration of HUVECs was detected by scratch test at 0, 12, 24 and 48 h. Scale: 50 μm. Magnification: × 100. (c, d) The protein levels of VEGF165 and VEGF165b were detected by ELISA. (e) The effect of HG on the tubule forming ability of HUVECs was detected. Scale: 50 μm. Magnification: × 100. (f-h) Western blot was used to assess the levels of Wnt5a, p-JNK1/JNK1, p-JNK2/JNK2 and p-JNK3/JNK3. *P < 0.05, **P < 0.01, ***P < 0.001.

## SFRP5 regulated the behavior and angiogenesis of HUVECs

As the circulating levels of SFRP5 correlate with impaired-glucose regulation in T2DM [34], we investigated the role of SFRP5 in regulating HUVECs activity and angiogenesis subsequently. Firstly, the level of SFRP5 was detected after HUVECs cells were cultured for 72 h at 30 mmol/L HG. Western blot results showed that the expression of SFRP5 was down regulated in HG group, which was compared with NC group (*P* < 0.05, Figure 2(a)). Then, the role and related mechanism of SFRP5 in regulating HUVECs cell proliferation, migration, and lumen formation were detected. SFRP5 interference and overexpression plasmid vector was constructed and transferred into the HUVECs model damaged by HG. At the same time, JNK inhibitor (sp600125) was added to the model cells transfected with plasmid, and the transfection efficiency was detected by qRT-PCR. Compared with NC group, the SFRP5 mRNA level in HG group was dramatically decreased, and the SFRP5 expression level in SFRP5 interference group and SFRP5 overexpression group were down-regulated and up-regulated, respectively, compared with HG group, however, the SFRP5 level was significantly up-regulated under the action of sp600125 (*P* < 0.05, Figure 2(b)). Western blot showed the same SFRP5 level (*P* < 0.05, Figure 2(g)). The results of cell scratch assay and tube forming ability assay showed that compared with HG group, the wound healing rate of HUVECs in SFRP5 interference group decreased, and the length of pipe network, nude, and tube decreased. However, the migration distance of HUVECs and the length of tube and nude increased in SFRP5 overexpression group. Sp600125 further promoted the role of SFRP5 in promoting HG induced HUVECs migration and angiogenesis (*P* < 0.05, Figure 2(c, d)). Likewise, ELISA confirmed that SFRP5 overexpression and deletion down-regulated and up-regulated the level of VEGF165, respectively. SP600125 enhanced the effect of SFRP5, while the level of VEGF165b showed the opposite result (*P* < 0.05, Figure 2(e, f)). Subsequently, we explored the Wnt5a/JNK pathway involved in SFRP5 regulation of HUVECs behavior and angiogenesis. Western blot showed that in HUVECs, the expression of Wnt5a, p-JNK1/JNK1, p-JNK2/JNK2, p-JNK3/JNK3 was downregulated and upregulated in SFRP5 interference group and SFRP5 overexpression group. However, under the action of SP600125, the expressions of Wnt5a, p-JNK1/JNK1, p-JNK2/JNK2, p-JNK3/JNK3 were substantially declined compared with HG group (*P* < 0.05, Figure 2(g)). This indicates that SP600125 enhances the downregulation of Wnt5a/JNK pathway protein by SFRP5, and that SFRP5 blocks Wnt5a/JNK pathway and promotes HUVECs migration and angiogenesis.

**Figure 2.** SFRP5 regulated the behavior and angiogenesis of HUVECs, 30 mmol/L HG was selected to act on HUVECs for 72 h, (a) The level of SFRP5 under HG was evaluated by Western blot. SFRP5 interference and overexpression plasmid vector was constructed and transferred into HG injured HUVECs model. At the same time, JNK inhibitor (sp600125) was added to the model cells transfected with plasmid, (b) The level of SFRP5 mRNA was detected by qRT-PCR. (c) The migration of HUVECs was detected by scratch test at 0, 12, 24 and 48 h. Scale: 50 μm. Magnification: × 100. (d) The tubule forming ability of HUVECs was detected by tubule forming ability experiment. Scale: 50 μm. Magnification: × 100. (e, f) The protein levels of VEGF165 and VEGF165b were detected by ELISA. (g) Western blot was used to assess the levels of SFRP5, Wnt5a, p-JNK1/JNK1,p-JNK2/JNK2 and p-JNK3/JNK3. *P < 0.05, **P < 0.01,***P < 0.001.

## SFRP5 inhibited cardiac dysfunction and promoted myocardial angiogenesis in T2DM-MI mice

Furthermore, the role of SFRP5 in myocardial infarction of type 2 diabetic mice was observed in vivo. Firstly, male C57 mice were fed with high-fat diet and intraperitoneal injection of streptozocin (STZ) for 3 days to establish T2DM model. The normal control group was injected with the same amount of citric acid buffer. After injection of STZ, fasting blood glucose of each mouse was measured for 3 consecutive days. Mice with blood glucose higher than 11.1 mmol/L were identified as T2DM mice. After T2DM model was established, MI model was established. Then, the cardiac function parameters of each group were measured by echocardiography. The results showed that CO, LVSF, and LVEF in T2DM and T2DM-MI mice were significantly lower than those in the control group. These results showed that the T2DM-MI mouse model was successfully established. Likewise, intervention with SFRP5 increased CO, LVSF, and LVEF levels. This suggests that SFRP5 inhibits cardiac dysfunction in T2DM-MI mice (*P* < 0.05, Figure 3(a-c)). Then, ELISA results showed that compared with the control group, VEGF165 was up-regulated, and VEGF165b was down regulated in T2DM group. T2DM + MI promoted the effect of T2DM. SFRP5 intervention down regulated VEGF165 and up regulated VEGF165b (*P* < 0.05, Figure 3(d, e)).

**Figure 3.** SFRP5 inhibited cardiac dysfunction and promotes myocardial angiogenesis in T2DM-MI mice T2DM + MI model was constructed *in vitro*. In T2DM + MI + SFRP5 group, SFRP5 (20 μg/kg*d) was injected intraperitoneally for 2 weeks. (a-c) Echocardiography was used to measure cardiac function parameters in each group, including CO, LVSF and LVEF. (d, f) The protein levels of VEGF165 and VEGF165b were detected by ELISA. *P < 0.05, **P < 0.01, ***P < 0.001.

## SFRP5 alleviated myocardial pathological injury and fibrosis in T2DM + MI mice

HE staining was performed to determine myocardial pathology (Figure 4a), and Masson staining was performed to depict the fibrotic area in the myocardium (Figure 4(b)). HE results showed that the muscle fibers in the control group were arranged orderly without other abnormalities. In T2DM group, a large number of inflammatory cells and fibrous hyperplasia appeared in the heart. Similarly, in T2DM + MI + vector group, we found uneven staining of cardiomyocytes, disordered arrangement of myocardial fibers, narrowed gap and obvious inflammation in necrotic area. In T2DM + MI + pcDNA-SFRP5 group, muscle fibers were arranged orderly and a small amount of inflammatory cells proliferated (Figure 4(a)). Likewise, Masson staining showed that the collagen fiber blue staining was more serious in T2DM and T2DM + MI + vector groups than in the control group. On the other hand, SFRP5 reduced collagen fibers compared with collagen fibers in T2DM + MI + vector group (Figure 4(b)). At the same time, SFRP5 treatment could down regulate the levels of caspase-3 and Bax and up regulate Bcl-2, indicating that SFRP5 could alleviate cardiomyocyte apoptosis in T2DM + MI mice. In addition, western blot results showed that compared with the control group, the expression of Wnt5a, p-JNK1/JNK1, p-JNK2/JNK2, p-JNK3/JNK3 in T2DM and T2DM + MI + vector groups increased, and SFRP5 down regulated the levels of Wnt5a, p-JNK1/JNK1, p-JNK2/JNK2, p-JNK3/JNK3 (*P* < 0.05, Figure 4(c)). This indicates that SFRP5 inhibits Wnt5a/JNK pathway and inhibits pathological damage and promotes myocardial regeneration in diabetic mice.

**Figure 4.** SFRP5 alleviated myocardial pathological injury and fibrosis in T2DM + MI mice. T2DM + MI model was constructed *in vitro*. In T2DM + MI + SFRP5 group, SFRP5 (20 μg/kg*d) was injected intraperitoneally for 2 weeks. (a) HE staining was used to determine myocardial pathology. Scale: 50 μm. Magnification: × 100. (b) Masson staining was used to depict the fibrotic area in the myocardium. Scale: 50 μm. Magnification: × 100. (c) The levels of SFRP5, Wnt5a, p-JNK1/JNK1, p-JNK2/JNK2, p-JNK3/JNK3, Caspase-3, Bax, Bcl-2 and TGF-β1.

## Discussion

Diabetes is one of the most common chronic diseases. In recent years, the number of diabetic patients has gradually increased. The main reason for the increase in the number of diabetic patients is population growth, aging, and lifestyle changes [35,36]. Diabetic neuropathy, including central nervous system and peripheral neuropathy, is one of the major complications of diabetes. In diabetic patients, the injury of cardiac sensory nerve fibers causes painless myocardial ischemia and increases the mortality of painless myocardial infarction in diabetics [37]. Previous studies have confirmed that SFRP5 plays a protective role in diabetic heart injury [19]. Impaired angiogenesis is the main cause of delayed wound healing in diabetes. Angiogenesis plays an important role in promoting the recovery of diabetic vascular complications [38]. Angiogenesis refers to the formation of new capillaries from preexisting blood vessels in the form of budding or non-budding through the proliferation and migration of vascular endothelial cells on the basis of original capillaries and/or venules. The process of angiogenesis is regulated by promoting angiogenesis factors and inhibiting angiogenesis factors, involving the proliferation, migration, tubule formation, and other cellular functions of endothelial cells [39]. Vascular endothelial growth factor (VEGF) is a multifunctional cytokine and an important factor in angiogenesis, including VEGF165 and VEGF165b [40,41].

In the current study, in order to simulate the model of hyperglycemia-induced injury to HUVECs, HUVECs were cultured in medium containing different concentrations of glucose for 24, 48, and 72 h, and the optimal HG concentration (30 mmol/L) was determined according to the lowest cell activity for 72 h for later functional experiments. Subsequently, the effects of SFRP5 on cell functions related to angiogenesis of HUVECs were studied, including cell migration and tubular structure formation, and the expression levels of and VEGF165 and VEGF165b were detected. We found that SFRP5 overexpression could improve the decreased mobility and lumen formation of HUVECs under HG and SFRP5 promoted the inhibitory effect of HG on angiogenesis. Futhermore, in this study, we constructed an isolated diabetic myocardial ischemic injury model to evaluate the effect and mechanism of SFRP5 on myocardial regeneration. It was found that SFRP5 could alleviate myocardial damage, pathological damage and fibrosis, and promote angiogenesis in diabetic mice with myocardial ischemia injury.

It has been reported that the inhibition of Wnt is involved in the angiogenesis of human umbilical vein [42–44]. Wnt5a, as one of the interacting binding proteins of SFRP5, has been reported to be involved in tumor progression [45,46], the above studies suggest that Wnt5a is involved in the process of angiogenesis and cell proliferation of a variety of cells, but there is no report on Wnt5a in vascular endothelium and vascular proliferation. Moreover, Gros et al. found that the non-classical Wnt signal Wnt5a/JNK plays an important role in the regulation of cell movement and cell division [47]. At the same time, a new study shows that Wnt5a/JNK3 is involved in the ischemia-reperfusion process of hippocampal CA1 area, and interfering with Wnt5a/JNK3 signaling pathway may provide a new way for the treatment of stroke [48], the above suggests that Wnt5a/JNK3 may be involved in the occurrence and development of cardiovascular diseases. However, whether Wnt5a/JNK3 is involved in angiogenesis and apoptosis of vascular endothelial cells has not been reported. In the current study, we assessed whether Wnt5a/JNK3 is involved in HG induced HUVECs angiogenesis and whether it plays a role in myocardial injury and angiogenesis in diabetic ischemic mice. The results showed that the expressions of Wnt5a, p-JNK1/JNK1, p-JNK2/JNK2, p-JNK3/JNK3 were significantly up-regulated in HG induced HUVECs and T2DM-MI mouse models, while SFRP5 down regulated the levels of Wnt5a, p-JNK1/JNK1, p-JNK2/JNK2, p-JNK3/JNK3. Under the action of JNK pathway inhibitor (SP600125), the expressions of Wnt5a, p-JNK1/JNK1, p-JNK2/JNK2, p-JNK3/JNK3 were significantly down regulated. This indicates that SFRP5 can promote the proliferation, migration and angiogenesis of HUVECs induced by HG through inhibiting Wnt5a/JNK signaling, and inhibit cardiac dysfunction, pathological damage, fibrosis, and myocardial angiogenesis in diabetic myocardial ischemia mice.

There are also some shortcomings in our experiments. First, we only explored SFRP5 to promote HG-induced HUVECs angiogenesis by inhibiting Wnt5a/JNK pathway, and to alleviate myocardial injury and promote myocardial angiogenesis in diabetic myocardial ischemia mice. This indicates that SFRP5 has other mechanisms in the protection of diabetic injury. In addition, although we provided the role of SFRP5 in HG induced HUVECs and diabetes mellitus combined with myocardial ischemic injury, specific clinical applications still needed corresponding clinical trials. In conclusion, SFRP5 plays a protective role in HG induced HUVECs and diabetes mellitus combined with myocardial ischemia. SFRP5 promotes HG induced HUVECs proliferation, migration and angiogenesis, and inhibits cardiac dysfunction, pathological damage, fibrosis, and myocardial angiogenesis by inhibiting Wnt5a/JNK signaling. The results of this study may provide new therapeutic targets for diabetic vascular complications.

## Conclusions

In summary, this study showed that significant effects of SFRP5 regulating on the angiogenesis and allevating MI as well as the downregulation of JNK signaling in HUVECs and T2DM mice with MI. Although the exact mechanisms underlying remain to be further clarified, our findings indicate a novel role for SFRP5 as a negative regulator in MI and support its potential role in the treatment of T2DM complicate with MI.

## Supplementary Material

Supplemental Material

## Data Availability

The data used to support the findings of this study are available from the corresponding author upon request.

## Abbreviations

T2DM: type 2 diabetes mellitus
SFRP5: secreted fizzled related protein 5
HUVECs: human umbilical vein endothelial cells
HG: High glucose
MI: myocardial infarction
VEGF: vascular endothelial growth factors
CO: cardiac output
LVSF: left ventricular shortening fraction
LVEF: left ventricular ejection fraction
JNK: c-Jun NH2-terminal Kinase
Wnt: wingless type
